RETRACTED

# Yanghe Decoction Effectively Alleviates Lung Injury and Immune Disorder in Asthmatic Mice Induced by Ovalbumin

**DOI:** 10.1155/2022/6040575

**Published:** 2022-05-05

**Authors:** Cui Li, Liming Tian, Yuwei Jiang, Yu Wang, Lingna Xue, Shaoyan Zhang, Xianwei Wu, Xing Huang, Lei Qiu, Zifeng Ma, Zhenhui Lu

**Affiliations:** Institute of Respiratory Disease, Longhua Hospital Shanghai University of Traditional Chinese Medicine, Shanghai 200032, China

## Abstract

**Objective:**

To probe into the ameliorative effect of Yanghe Decoction on pulmonary injury and immunologic derangement in asthmatic mice.

**Methods:**

C57BL/6 mice were randomized into control (Con), Model, and Yanghe Decoction (YHF) groups, with 12 in each. The asthma model of adult female mice was induced by ovalbumin in the Model group, and the YHF group was treated by Yanghe Decoction on the basis of asthma modeling. The Con group received the same amount of normal saline. Inspiratory resistance (Ri), expiratory resistance (Re), lung compliance (CL), and maximal voluntary ventilation (MVV) were measured after modeling. Lung tissue was collected for the measurement of interleukin (IL)-4, IL-5, IL-6, IL-10, IL-13, and tumor necrosis factor-*α* (TNF-*α*) by ELISA kits. Combined with HE staining and PAS staining, the pathological alterations of the lung in each group were observed, and CD4+, Th2, and Th1 contents were determined by flow cytometry (FCM).

**Results:**

The pulmonary function (PF) test revealed notably reduced Ri and Re as well as enhanced CL and MVV in asthmatic mice after the application of Yanghe Decoction. Yanghe Decoction dramatically ameliorated the pathological changes of lung tissue in asthmatic mice, as demonstrated by the staining results. ELISA results showed that Yanghe Decoction validly reduces lung tissue IL-4, IL-5, IL-6, IL-13, TNF-*α* and upregulates IL-10 in asthmatic mice. FCM indicated that Yanghe Decoction obviously reduced the number of Th1 and Th2 cells in asthmatic mice, although it caused the decrease of CD4+ cells, but the difference was not statistically significant.

**Conclusions:**

Yanghe Decoction can effectively ameliorate the inflammatory reaction, immune cell disorder, and PF injury in ovalbumin-induced asthmatic mice.

## 1. Introduction

Asthma is a chronic heterogeneous disease of the lower respiratory tract, which is clinically characterized by a chronic inflammatory response (IR) and airway hyper responsiveness, resulting in cough, wheezing, shortness of breath, and chest tightness [1]. The occurrence and development of asthma are complicated and involve multiple factors. At this stage, the pathogenesis of asthma cannot be completely defined, but the genome, environmental factors, and even early abnormal immune maturation may be the predisposing factors [2]. There are approximately 241 million asthma patients worldwide, as indicated by relevant statistics [3]. With advances in diagnosis and treatment, the prevalence of asthma has increased in recent years, especially in developing countries, while the mortality rate has decreased significantly [4, 5]. Asthma causes a grave physical and economic burden on patients and enormously reduces their daily life quality. However, the treatment of asthma still faces severe challenges. Chronic inflammation and airway remodeling are the two major causes of asthma attacks. In the progression of asthma, the IR caused by immunologic derangement exacerbates the degree of airway stenosis, which leads to airway remodeling in cooperation with airway thickening, leading to significant respiratory obstruction and progressive decline in pulmonary function (PF) [6, 7]. At this stage, asthma treatment focuses on improving inflammation, which cannot fundamentally ameliorate the PF injury and prevent the disease from worsening [7]. Hence, the current asthma treatment strategy should center on the joint amelioration of pulmonary injury and immunologic derangement in asthma patients.

RETRACTED

Accumulating studies have confirmed that traditional Chinese herbal medicine is helpful for asthma, antiinflammatory, and antipulmonary injury management. A randomized double-blind trial [8] showed that Pingchuan Yiqi Granule (a traditional Chinese medicine [TCM] formula) can validly ameliorate the pulmonary dysfunction of asthma patients and reduce inflammatory factors (IFs) interleukin (IL)-5, IL-8, IL-1*β*, and PGD2. TCM-assisted therapy can partly improve the clinical effect of conventional treatment strategies on children with asthma [9]. We have previously reported the therapeutic effect of Jia-Wei-Yu-Ping-Feng-San on asthmatic mice [10], and in this study, we will provide another new method of treating asthmatic mice with traditional Chinese herbal medicine: Yanghe Decoction. The main components of Yanghe Decoction include Rehmannia glutinosa, Colla Cornus Cervi, Cinnamomum cassia, Ephedra sinica, Semen Sinapis, Rhizoma Zingiberis Preparata, and Glycyrrhiza. Yanghe Decoction has been proved to play a significant antiinflammatory role in disease treatment through the NLRP3 inflammatory inflammasome [11], as well as JAK/STAT [12] and Wnt/*β*-catenin [13] pathways. It is worth noting that Yanghe Decoction has great potential therapeutic value in asthma treatment. A study [14] pointed out that TCM granules based on Yanghe Decoction may meliorate the IR and bronchial lesions in asthmatic mice through the PI3K axis.

RETRACTED

At present, there are few studies on treating asthma with Yanghe Decoction. To investigate the application value of Yanghe Decoction in asthma treatment, this study adopted the ovalbumin-induced asthma mouse model and administration of Yanghe Decoction, combined with enzyme-linked immunosorbent assay (ELISA), flow cytometry (FCM), pathological staining, and PF detector, to explore the amelioration effect of Yanghe Decoction on PF and immune function of asthmatic mice. The new findings of this research will provide reliable basic experimental data for the clinical application of Yanghe Decoction in the treatment of asthma, and expand the treatment prospects of TCM in modern medicine.

## 2. Materials and Methods

### 2.1. Animals

Six-week-old female C57BL/6 mice (Vital River Experimental Animal Technology, Beijing, China) weighed 18–20 g and were allowed to eat and drink freely under alternated 12 hours of light/darkness. All animals were reared at a constant temperature (25 ± 1 °C) and humidity (50%). The hospital ethics committee ratified this research without reserves. All animal experimental operations were strictly in compliance with the Guidelines for the Care and Use of Laboratory Animals [15].

### 2.2. The Model of Ovalbumin-Induced Asthma

The mice were randomized into control (Con), model, and YHF groups, with 12 in each. The model and YHF groups received ovalbumin (OVA) to induce asthma. The induction, which was divided into two stages: sensitization and stimulation, lasted for 28 days, with the day of the first induction recorded as day 0. Sensitization: 0.1 mL OVA-aluminum hydroxide solution (1 mg/mL) was injected intraperitoneally on day 0 and 7, respectively. Stimulation: from days 14–22, mice were challenged with a 3% aerosolized OVA solution through an ultrasonic nebulizer for 30 min every other day, followed by an intranasally installed 50 µl dose of 1 mg/ml OVA (total 50 µg) daily on days 24, 25, and 26. Mice in the Con group were sensitized and challenged with saline. While those in the YHF group received Yanghe Decoction on day 14, a solvent made of powder (1.47 g/kg) was administered by gavage once a day for 14 days. The administration of Yanghe Decoction was completed 30 min before atomization. The granules of Yanghe Decoction, with the main ingredients of Prepared Colla Cornus Cervi (9 g), Cinnamomum Cassia (3 g), Dried Ginger Charcoal (2 g), Chinese Ephedra (2 g), Semen Brassicae (6 g), Raw Licorice (3 g), and Rehmannia glutinosa (30 g), were obtained from Longhua hospital and mixed according to the dose recommended by the doctors. The Chinese medicine granules were dissolved in sterile water and then administered to the animals by gavage.

RETRACTED

### 2.3. PF Test

On day 28, mice were injected with 1% of pentobarbital sodium intraperitoneally after atomization induction. Then, they were placed on their backs in the closed box of small animal ventilators and intubated. The inspiratory resistance (Ri), expiratory resistance (Re), lung compliance (CL), and maximal voluntary ventilation (MVV) were measured.

### 2.4. FCM

Part of the lung tissue was cut into 3 cm × 2 cm pieces, which were digested by type IV collagenase at 37 for 3 h. CD4 + T cells were identified by CD3+CD8-cells after obtaining the cell suspension. In brief, phorbol myristate acetate (PMA) solution (to activate T cells) and ionomycin solution (to inhibit cytokine secretion) incubated the cell suspension together at 37 °C for 4 h. Then, CD3-PC5 and CD8-FITC antibodies were placed in the samples for incubation for a certain period of time. Intraprep permeabilization reagent was used to fix and break the film. Then, IL-4-PE (for determining Th1) and IFN-*γ*-PE (for determining Th2) antibodies were added to the samples. After PBS washing and resuspension, the precipitation was detected on the machine. CD4+, Th1, and Th2 cells were counted. IL-4-PE and IFN-*γ*-PE antibodies were offered by R & D Systems, USA, while CD3-PC5 and CD8-FITC antibodies were provided by Beckman Coulter, USA.

### 2.5. ELISA

Lung tissue samples were collected for ELISA. A 96-well plate was added to the coating solution for coating treatment. Then, the cell supernatant sample was diluted and added into the coated reaction well and immersed in biotin antibody working solution, enzyme conjugate working solution, TMB substrate solution, and 2M sulfuric acid in turn according to the requirements of the instructions. The absorbance was measured at a 450 nm wave peak with a microplate reader, and the contents of IL-4, IL-5, IL-6, IL-10, IL-13, and tumor necrosis factor-*α* (TNF-*α*) were calculated according to the standard curve. The above ELISA kits were all provided by Abcam.

### 2.6. Pulmonary Pathology Observations

Following immobilization with 10% formalin, the lung tissue was dehydrated with alcohol, made transparent with xylene, embedded with wax, sliced, and dried at 45. During dyeing, xylene was added for dewaxing, and the slices were soaked in high-to-low-concentration alcohol, followed by the addition of distilled water to restore moisture. HE staining and PAS staining were added for a certain time, and then, the lung tissue was dehydrated, transparent, and sealed for the observation of pathological changes under a light microscope. HE and PAS kits were offered by Shanghai Beyotime Biotech.

### 2.7. Statistics and Analysis

The experiment was run in triplicate, and the measurement results were given as Mean ± SEM. The difference between the data was analyzed by SPSS 20.0 (USA), and the image rendering was performed by Graphpad 8.0. Differences among multiple groups were analyzed by one-way analysis of variance, and post-hoc pairwise comparisons were made by the LSD-t-test. All comparisons were two-tailed. With 95% as its confidence interval, a statistically significant difference was assumed at *P* < 0.05.

RETRACTED

## 3. Results

### 3.1. Impact of Yanghe Decoction on PF of Asthmatic Mice

In this study, the differences of PF indexes, such as Ri, Re, CL, and MVV, were analyzed with the ventilator, with the results presented in Figure 1. The Model group had noticeably elevated Ri and Re while remarkably reducing CL and MVV than Con group. While in comparison with the Model group, YHF effectively reduced Ri and Re and ameliorated CL and MVV of asthmatic mice. The results indicate that Yanghe Decoction can validly improve the PF parameters of asthmatic mice.

YHF denotes Yanghe Decoction. ^^*∗∗∗*^^ indicates *P* < 0.001 and ### indicates *P* < 0.001 vs. the Model group.

### 3.2. Impact of Yanghe Decoction on IR in Asthmatic Mice

In this study, lung tissue IFs IL-4, IL-5, IL-6, IL-10, IL-13, and TNF-*α* in asthmatic mice were detected by ELISA, with the results shown in Figure 2. Asthma caused the lung tissue IL-4, IL-5, IL-6, IL-13, and TNF-*α* obviously increase, while IL-10 notably decreased, indicating that asthmatic mice were in an obvious inflammatory state. Compared with the Model group, Yanghe Decoction effectively reduced IL-4, IL-5, IL-6, IL-13, and TNF-*α* and upregulated IL-10. This result indicates that Yanghe Decoction can effectively alleviate the IR in asthmatic mice.

### 3.3. Impact of Yanghe Decoction on Immune Function of Asthmatic Mice

Herein, the number of CD4+, Th1, and Th2 cells was measured by FCM, and the results are shown in Figure 3. The significant increase of CD4+, Th1, and Th2 cell numbers indicated ovalbumin-induced Th1 and Th2 cell responses in mice. Yanghe Decoction statistically reduced Th1 and Th2 cell numbers in asthmatic mice. Although the YHF group had fewer CD4+ cells than the Model group, the difference was not remarkably significant.

### 3.4. Impact of Yanghe Decoction on Pathological Changes of Lung Tissue in Asthmatic Mice

In this study, HE staining and PAS staining were used to determine the pathological changes in the lung tissue of mice in each group, and the results are shown in Figure 4 and 5. HE staining showed bronchitis inflammatory cell infiltration and partial bronchial mucus formation in asthmatic mice, while Yanghe Decoction obviously ameliorated inflammation infiltration and mucus formation induced by asthma (Figure 4). In addition, PAS staining results showed obvious goblet cell metaplasia of airway epithelium in asthmatic mice, which was effectively alleviated by Yanghe Decoction (Figure 5). These results suggest that Yanghe Decoction can effectively ameliorate airway inflammation and airway remodeling caused by asthma.

RETRACTED

## 4. Discussion and Conclusion

TCM is characterized by fewer side effects and lower economic costs. The latest evidence shows that TCM-assisted therapy based on Yanghe Decoction is one of the most common adjuvant therapy schemes for antimalignant tumor treatment. A previous study [16] reported that Yanghe Decoction inhibited angiogenesis and epithelial-mesenchymal transition of human epidermal growth factor receptor 2 (HER2) positive breast cancer through the Akt pathway. Besides the remarkable part of Yanghe Decoction in anticancer management, it also plays an effective antiinflammatory part in the progression of some diseases. The main components of Yanghe Decoction, such as Glycyrrhiza uralensis Fisch [17] and Cinnamomum cassia [18, 19], have been proved to obviously alleviate disease inflammation. A clinical study [20] reported the amelioration effect of Yanghe Decoction on patients with ankylosing spondylitis, suggesting that Yanghe Decoction has potential clinical application value in ameliorating autoimmune diseases.

A study [14] indicates that Chinese medicinal granules based on Yanghe Decoction may ameliorate the IR of asthmatic mice through the PI3K pathway, on which basis we found that Yanghe Decoction remarkably reduced the content of IFs, CD4+, Th1, and Th2 in asthmatic mice. Asthma is an autoimmune disease in which inflammation and immune cell disorders are the main causes. From the results of this study, Yanghe Decoction seems to alleviate asthma inflammation by regulating immune cells. The increase of Th1 cells in asthmatic mice leads to the synthesis and secretion of IFs in vivo, while Th2 senses IR and responds to suppress excessive IR [21]. Notably, we observed that IL-10 was reduced in asthmatic mice, but its level was restored by treatment with Yanghe Decoction. IL-10 is an important inflammatory suppressor, so the decrease of IL-10 will markedly promote asthmatic mice to be in a proinflammatory state, while Yanghe Decoction may achieve its antiinflammatory effect by inducing the production of IL-10. Yanghe Decoction can improve the immune function of asthmatic mice and inhibit Th1 cell-mediated IR, thus further alleviating Th2 cell disorder. We also observed that the lung tissue of OVA-induced asthmatic mice showed inflammatory cell infiltration around the bronchus and partial bronchial mucus formation, which greatly deteriorated the lung function of mice, while Yanghe Decoction effectively mitigated the pulmonary injury of the asthmatic mice. The lung damage associated with asthma arises from an autoinflammatory state. IR leads to significant pathological changes in respiratory epithelial tissue, thus promoting airway remodeling in asthma [22]. Therefore, the antiinflammatory effect of Yanghe Decoction regulates inflammation-dependent airway remodeling, thus relieving the degree of pulmonary injury in asthmatic mice.

RETRACTED

### 4.1. Limitation and Future Work

Although this research combined with an OVA-induced asthma animal model to verify the amelioration effect of Yanghe Decoction on the lung and immune function of asthmatic mice, the specific molecular mechanism involved still needs to be further explored by combining cellular models such as airway smooth muscle cells, vascular endothelial cells, and fibroblasts around the airway.

To sum up, this study suggests that Yanghe Decoction can effectively alleviate the lung dysfunction of OVA-induced asthma mice, relieve the inflammatory state in mice, and inhibit immunologic derangement. This study provided reliable scientific research data for the clinical application of Yanghe Decoction and qualified the improvement effect of Yanghe Decoction on lung and immune functions in asthma. However, the potential mechanism of Yanghe Decoction in asthma treatment still needs further study, combined with *in vivo/in vitro* models.

## Figures and Tables

**Figure 1:** Lung function indexes of mice in each group (*n* = 12). (a) Inspiratory resistance (Ri). (b) Expiratory resistance (Re). (c) Lung compliance (CL). (d) Maximum ventilation volume (MVV).

**Figure 2:** Effect of Yanghe Decoction on lung tissue inflammatory factors in asthmatic mice (*n* = 12). (a) Interleukin-4 (IL-4). (b) Interleukin-5 (IL-5). (c) Interleukin-6 (IL-6). (d) Interleukin-10 (IL-10). (e) Interleukin-13 (IL-13). (f) Tumor suppressor factor-*α* (TNF-*α*). ^*∗∗∗*^ indicates *P* < 0.001 *vs.* the control group and ### indicates *P* < 0.001 *vs.* the Model group.

**Figure 3:** Effect of Yanghe Decoction on immune function of asthmatic mice (*n* = 12). (a) CD4+ cell number; (b) TH2 cell number; and (c) TH1 cell number. ^*∗*^indicates *P* < 0.05, ^*∗∗*^indicates *P* < 0.01, and ^*∗∗∗*^indicates *P* < 0.001 vs the control group. NS indicates *P* > 0.05, ^#^indicates *P* < 0.05, ^##^indicates *P* < 0.01, and ^###^indicates *P* < 0.001 *vs* the Model group.

**Figure 4:** Observation of the effect of Yanghe Decoction on the pathological changes of lung tissue in asthmatic mice based on HE staining (*n* = 12, 200X). YHF denotes Yanghe Decoction.

RETRACTED

**Figure 5:** Observation of the effect of Yanghe Decoction on the pathological changes of lung tissue in asthmatic mice based on PAS staining (*n* = 12, 200X). YHF denotes Yanghe Decoction.

## Data Availability

The simulation experiment data used to support the findings of this study are available from the corresponding author upon request.

## Additional Points

*Challenges in Data Collection*. In the domain of medical and healthcare, the availability of data publically remained a challenge till date [23–26]. Therefore, we turned towards our own experimentation and data collection.
